The article "Design of Optimum Portfolio Scheme Based on Improved NSGA-II Algorithm" was published in 2022. Journal: Comput Intell Neurosci.

# Design of Optimum Portfolio Scheme Based on Improved NSGA-II Algorithm

**DOI:** 10.1155/2022/7419500

**Published:** 2022-06-13

**Authors:** Yiqian Zhou, Weinan Chen, Deqin Lin

**Affiliations:** ^1^Faculty of Business, City University of Macau, Macau 999078, China; ^2^Faculty of Finance, City University of Macau, Macau 999078, China

## Abstract

In the financial industry, it is of great significance to study the multiobjective portfolio optimization for obtaining a reasonable investment strategy. This paper designs the financial portfolio scheme based on the multiobjective optimization algorithm that is based on the framework of the NSGA-II algorithm. In order to introduce convergence information, aiming at the actual problem of the portfolio, the mixed individual coding mechanism with asset information expands the application of the multiobjective evolutionary algorithm in portfolio optimization. The portfolio scheme obtained is effective, which is helpful to improve the decision-making efficiency of financial investors and enriches the application of modern financial theory.

## 1. Introduction

With the rapid development of the financial market, investment and financial management are no longer limited to a single way of saving with more investments in securities. How to use more scientific and rational investment strategies to realize capital appreciation has become a problem that investors must consider and pay attention to. Generally speaking, the purpose of investment and financial management is to maximize the income, but benefits and risks often exist at the same time. A portfolio can spread risks, and the key lies in how to allocate assets and how to deal with the relationship between risks and benefits.

At present, the financial industry, as one of the important components of China's economy, has been widely concerned by people in various fields. In reality, the investment fields and fund types are complicated, so the essence of designing a relatively optimal portfolio is a high-dimensional multiobjective optimization problem [1–4]. Meanwhile, the heuristic algorithm can get a satisfactory solution in polynomial time, such as evolutionary algorithm, simulated annealing algorithm, artificial neural network, and quantum algorithm [5–7]. Because of the inherent multiobjective nature of portfolio problem, many scholars usually use a multiobjective evolutionary algorithm to solve it, such as weighting method, constraint method, objective programming method, and minimax method. A multiobjective optimization algorithm does not need to obtain the derivative information of the problem nor does it need to aggregate optimization objectives with different properties. It can deal with enormous scope search space autonomously, where the problem can be solved by parallel search of cyclic iteration, and the average fitness of the species is improved generation by generation to approach the global optimal solution [8, 9]. Therefore, the customized improvement of the problem model can not only expand its related research but also help to advance the decision-making efficiency of investors.

The article "Design of Optimum Portfolio Scheme Based on Improved NSGA-II Algorithm" was published in 2022. Journal: Comput Intell Neurosci.

## 2. Theoretical Basis of Portfolio

With the rapid development of science and technology and the continuous improvement of the financial system, China's financial market is actively integrated with foreign countries where financial products are becoming more diversified, and bonds, stocks, futures, foreign exchange, and various Internet financial derivatives are gradually moving towards the investment scope of ordinary people [10]. Investment is the act of converting funds into assets or capital in a certain period of time, so as to obtain economic returns or value-added benefits. No matter what kind of investment is made, the purpose is to obtain higher returns. However, benefits and risks often coexist. Investors want to get as many benefits as possible and at the same time bear as little risk as possible. Therefore, how to maintain and increase the value of assets through investment and financial management is a great challenge.

### 2.1. Single Investment

The quantitative relationship is applied to the research of portfolio theory, the benefits and risks are quantified, and the two goals of maximizing benefits and minimizing risks are put forward to solve the problems of selection of financial products and allocation of capital proportion for investors [11, 12].

In actual investment activities, the average historical real rate of return is usually used to replace the expected rate of return to measure the pros and cons of the portfolio. Assuming that there are *M* securities in the securities pool, the actual rate of return of securities is calculated as shown in the following formula:

(1) $$\begin{array}{c} r_{i}=\frac{S_{i}\left(t\right)-S_{i}\left(0\right)}{S_{i}\left(0\right)}, \end{array}$$

where *r*_*i*_ is the actual rate of return of a security, *S*_*i*_(*t*) is the closing price of the securities at the end of the holding period, and *S*_*i*_(0) is the closing price of the securities at the initial stage of the cycle.

The company's operation and performance usually have certain stability; therefore, the average historical actual rate of return can be used as the estimate of the expected rate of return of the securities. Assuming that vector *R*_*i*_=(*r*_*i*_^1^, *r*_*i*_^2^,…,*r*_*i*_^*T*^)^*T*^ represents the vector composed of multiperiod historical return rate of the ith asset, so the expected return rate is shown in the following formula:

(2) $$\begin{array}{c} \bar{R_{i}}=E\left(R_{i}\right)=\sum_{t=1}^{T}r_{i}^{t}p_{i}^{t}, \end{array}$$

where ${\bar{R}}_{i}$ is the expected return on a security, *T* is the number of periods with the historical real return, *r*_*i*_^*t*^ is the real return on the security in term *t*, and *p*_*i*_^*t*^ is the probability that the real return is *r*_*i*_^*t*^.

The article "Design of Optimum Portfolio Scheme Based on Improved NSGA-II Algorithm" was published in 2022. Journal: Comput Intell Neurosci.

In investment activities, it is uncertain to use the historical rate of return to estimate the expected rate of return because the real return may be higher than expected or lower than expected, which is the risk faced by many investors. Therefore, the risk needs to be quantified by the variance of the expected rate of return. For a single security, the risk can be calculated by the following formula:

(3) $$\begin{array}{c} \sigma^{2}=D\left(R_{i}\right)=\sum_{t}^{T}{\left(r_{i}^{t}-\bar{R_{i}}\right)}^{2}p^{t}. \end{array}$$

The above formula uses the volatility of security returns; that is, the variance *σ*^2^ of the expected return rate of a security is adopted to quantify the risk. The larger the variance is, the greater the deviation between the actual return rate and the expected return rate is, which indicates that the returns of security are highly uncertain, and the investment risk is strong.

### 2.2. Portfolio Investment

Assuming a portfolio chooses N sorts of resources from the protections pool and joins them as indicated by a specific venture proportion, then in a certain investment cycle, the pay of the portfolio is measured by the weighted normal amount of the return paces of every resource, which can be calculated by the following formula:

(4) $$\begin{array}{c} r_{p}=\sum_{i=1}^{N}x_{i}\bar{R_{i}}, \end{array}$$

where *r*_*p*_ represents the expected return rate of the portfolio and *x*_*i*_ represents the proportion of the ith asset in the portfolio, which meets the budget constraint ∑_*i*=1_^*N*^*x*_*i*_=1, $x_{i}>0,\bar{R_{i}}$.

In the actual market, all kinds of securities are not completely independent, and there are always some connections. This correlation between securities is usually expressed by covariance, which is the expectation to measure the overall error between two variables [13]. In the actual portfolio, investors usually want to choose some unrelated assets as far as possible to spread the risk as much as possible, so set *R*=(*R*_1_, *R*_2_,…,*R*_*N*_)^*T*^ as the actual rate of return of each security in the portfolio, and the covariance between *i* and *j* securities is calculated by the following formula:

(5) $$\begin{array}{c} \sigma_{ij}=\mathrm{cov}\left(R_{i},R_{j}\right)\\ =\frac{1}{T}\sum_{t}^{T}\left(r_{i}^{t}-\bar{R_{i}}\right)\left(r_{j}^{t}-\bar{R_{j}}\right). \end{array}$$

Using variance *σ*_*p*_^2^ as a measure of portfolio risk, we should consider not only the characteristics of individual securities but also the relationship between them. The portfolio risk is expressed by the following formula:

(6) $$\begin{array}{c} \sigma_{p}^{2}=D\left(R\right)\\ =\sum_{i}^{N}\sum_{j}^{N}x_{i}y_{j}\sigma_{ij}. \end{array}$$

The article "Design of Optimum Portfolio Scheme Based on Improved NSGA-II Algorithm" was published in 2022. Journal: Comput Intell Neurosci.

## 3. Multiobjective Optimization Algorithm

### 3.1. Algorithm Design

NSGA-II algorithm is a far-reaching multiobjective optimization algorithm at present. Since it was put forward, because of its simplicity and high efficiency, this algorithm has become one of the basic algorithms in problems of multiobjective optimization [14]. As shown in Figure 1, the main advantages of this algorithm compared with traditional NSGA are as follows.

1. The fast nondominated sorting algorithm reduces the computational complexity from the original mN^3^ to mN^2^, where *n* is the species size and *m* is the quantity of goal capacities.
2. The addition of the crowding degree and crowding degree comparison operator not only solves the shortcoming of artificial designation of shared parameters in the algorithm but also enables the species to be homogeneously extended to the whole Pareto domain through crowding degree, thus ensuring the diversity of the species.
3. Introduction of elite strategy and expansion of sampling space combine the parent and the offspring together to produce the next generation of the species by competition is beneficial to preserve the excellent individuals of the previous generation of the species. At the same time, the stratified storage of individuals in the species reduces the loss of the best individuals, improves the overall level of the species, and greatly optimizes the accuracy of the algorithm.

The NSGA-II algorithm adopted in this paper can improve the diversity of the species and make the level of the species improve rapidly. The flow chart of the algorithm is shown in Figure 2.

1. Initialize the species and set its size as *n*, after the nondominated sorting of the species with the size of *n*, execute the traditional genetic algorithm, and obtain the first-generation progeny species through crossover, mutation, and selection
2. Combine the parent and offspring species into a species, calculate the crowding degree of individuals in the nondominant layer simultaneously through rapid nondominant sorting, and select suitable individuals to form a new parent species by using crowding degree and nondominant relationship
3. Generate a new progeny species through the basic operations of crossover, mutation, and selection in a traditional genetic algorithm, and repeat the above steps until the maximum number of iterations is met

The article "Design of Optimum Portfolio Scheme Based on Improved NSGA-II Algorithm" was published in 2022. Journal: Comput Intell Neurosci.

### 3.2. Optimized Algorithm

t-SNE algorithm is introduced to reduce the problem of target redundancy in high-dimensional multitargets, which greatly decreases the running time and the load of devices and improves the accuracy of the algorithm. The flow chart is shown in Figure 3.

Firstly, the original target set *I*_0_ was selected to initialize the species, and then, the NSGA-II algorithm was performed to optimize the species to form a new parent species *P*_0_. Then, t-SNE algorithm is optimized for *P*_0_ to obtain the nonredundant target set *I*_1_. Finally, the above steps are repeated until the maximum number of iterations is satisfied, and the species *P*_2_, *P*_3_,…*P*_*t*−2_*P*_*t*−1_, and target set *I*_3_,…, *I*_*t*_, when *I*_*t*−1_=*I*_*t*_, the Pareto optimal solution *P*_*t*−1_ of the target set can be obtained.

### 3.3. Implementation Process of Algorithm

Assuming that the number of targets is *N*, the target set is *I*_*t*_, and gen is the number of iterations.

(1) Set *t*=0, the initial target set is *I*_0_={1,2,…, *N*}, and then, the species of the target set is initialized. *P*, where selection, suitable individuals are selected to form a new parent species *P*_0_ by fast nondominated sorting and calculating crowding degree. The binary crossover can be simulated as follows:
  (7) $$\begin{array}{c} x_{1j}\left(t\right)=0.5*\left[\left(1+\gamma_{j}\right)x_{1j}\left(t\right)+\left(1-\gamma_{j}\right)x_{2j}\left(t\right)\right],\\ x_{2j}\left(t\right)=0.5*\left[\left(1+\gamma_{j}\right)x_{1j}\left(t\right)+\left(1-\gamma_{j}\right)x_{2j}\left(t\right)\right]. \end{array}$$
Among them,
  (8) $$\begin{array}{c} \gamma_{j}=\left\{\begin{array}{cc} {\left(2u_{j}\right)}^{1/\left(n+1\right)}, & u_{j}<0.5,\\ {\left(\frac{1}{2\left(1-u_{j}\right)}\right)}^{1/\left(\eta +1\right)}, & \text{else.} \end{array}\right) \end{array}$$
(2) Calculate the pairs of Euclidean distances between samples of *P*_0_ species, and calculate the joint probability *p*_*ij*_ between pairs of data points in high-dimensional space.
  (9) $$\begin{array}{c} p_{ij}=\frac{p_{j|i}+p_{i|j}}{2n}, \end{array}$$
   where *δ*_*i*_ represents the variance of the Gaussian function centered on the data point, *x*_*i*_ represents the initial population characteristic matrix, and *p*_*ji*_ represents the conditional probability of similarity between the data point *x*_*i*_ and data point *x*_*j*_ of the species characteristic matrix.
  (10) $$\begin{array}{c} p_{j|i}=\frac{\exp\left(-x_{i}-x_{j}^{2}/2\delta_{i}^{2}\right)}{\sum_{k\neq i}\exp\left(-x_{i}-x_{k}^{2}/2\delta_{i}^{2}\right)}. \end{array}$$
(3) Calculate joint probability *q*_*ij*_ between low dimensional spatial data point pairs in *P*_0_ Eigenmatrix.
  (11) $$\begin{array}{c} q_{ij}=\frac{{\left(1+y_{i}-y_{j}^{2}\right)}^{-1}}{\sum_{k\neq l}{\left(1+y_{l}-y_{k}^{2}\right)}^{-1}}, \end{array}$$
   where *y*_*i*_, *y*_*j*_, *y*_*l*_, and *y*_*k*_ represent the data point of the species characteristic matrix.
(4) Calculate the KL divergence between *p*_*ij*_ and *q*_*ij*_, and work out the objective function *C*:
  (12) $$\begin{array}{c} C=\text{KL}\left(P\left\|\right)Q\right)=\sum_{i}\sum_{j}p_{ij}\log\frac{p_{ij}}{q_{ij}}. \end{array}$$
(5) Solve the gradient of *P* and *Q*:
  (13) $$\begin{array}{c} \frac{\delta C}{\delta y_{i}}=4\sum_{j}\left(p_{ij}-q_{ij}\right)\left(y_{i}-y_{j}\right){\left(1+y_{i}-y_{j}^{2}\right)}^{-1}. \end{array}$$
(6) Get the target set *I*_1_, and repeat (1) ∼ (5) until the set maximum iteration algebra is met, and the species is obtained. *P*_2_, *P*_3_,…, *P*_*t*−2_, *P*_*t*−1_ and target set *I*_3_,…, *I*_*t*_, when *I*_*t*−1_=*I*_*t*_, and find the Pareto optimal solution of the target set *P*_*t*−1_.
Calculate the target set *I*_1_, and repeat step (1) ∼ (5) until the maximum iteration algebra is satisfied, and the species *P*_2_, *P*_3_,…, *P*_*t*−2_, *P*_*t*−1_ and target set *I*_3_,…, *I*_*t*_, when *I*_*t*−1_=*I*_*t*_, the Pareto optimal solution *P*_*t*−1_ of the target set can be obtained.

The article "Design of Optimum Portfolio Scheme Based on Improved NSGA-II Algorithm" was published in 2022. Journal: Comput Intell Neurosci.

## 4. Multiobjective Portfolio Model

### 4.1. Problem Description

The financial market has many nonrandom factors, such as fuzziness and uncertainty. Therefore, this paper tries to express the fuzzy uncertainty of the financial market with fuzzy theory. Investors usually refer to financial intermediaries. The main reason why diversified investment reduces the risk is that the correlation of different types of companies is poor or even negative. After the formation of the portfolio, the correlation of the portfolio is dissolved, so that the variance of the portfolio decreases; that is, the risk decreases. In investment theory, diversified investment is common that it can effectively reduce risks [17, 18]. Based on the fuzzy theory, a profit-risk optimization model is established with constraints, where the profit and risk are regarded as two optimization objectives in the model.

Assuming that *R* represents all real numbers, A is the convex fuzzy number defined on *R* with continuous membership function *μ*_*A*_(*x*), and F is the whole fuzzy set defined on the real number field *R*.

**Definition 1 .**

The article "Design of Optimum Portfolio Scheme Based on Improved NSGA-II Algorithm" was published in 2022. Journal: Comput Intell Neurosci.

Assume $A\in F,{\left[A\right]}_{\gamma }=\left[a\left(\gamma \right),\bar{a}\left(\gamma \right)\right]\left(\gamma \in \left[0,1\right]\right)$, and *A* represents the *γ*-horizontal cut set, then the probability mean of fuzzy number *A* is defined as

(14) $$\begin{array}{c} E\left(A\right)=\int_{0}^{1}\gamma \left(\underline{a}\left(\gamma \right)+\bar{a}\left(\gamma \right)\right){\text{d}}_{\gamma },\\ \text{Var}\left(A\right)=\int_{\text{0}}^{1}\gamma \left[{\left(E\left(A\right)-\underline{a}\left(\gamma \right)\right)}^{2}+{\left(E\left(A\right)-\bar{a}\left(\gamma \right)\right)}^{2}\right]{\text{d}}_{\gamma }. \end{array}$$

Lower half probability variance of *A* is

(15) $$\begin{array}{c} {\text{Var}}^{-}\left(A\right)=2\int_{0}^{1}\gamma {\left(E\left(A\right)-\underline{a}\left(\gamma \right)\right)}^{2}{\text{d}}_{\gamma }. \end{array}$$

Upper half probability variance of *A* is

(16) $$\begin{array}{c} {\text{Var}}^{+}\left(A\right)=2\int_{0}^{1}\gamma {\left(E\left(A\right)-\bar{a}\left(\gamma \right)\right)}^{2}{\text{d}}_{\gamma }. \end{array}$$

If *A*=(*a*, *b*, *α*, *β*) is A trapezoidal fuzzy number, its membership function *μ*_*A*_(*x*) is shown in Figure 4.

(17) $$\begin{array}{c} \mu_{A}\left(x\right)=\left\{\begin{array}{cc} \frac{x-\left(a-\alpha \right)}{\alpha }, & a-\alpha \leq x\leq a,\\ 1, & a\leq x\leq b,\\ \frac{b+\beta -x}{\beta }, & b\leq x\leq b+\beta ,\\ 0, & \text{else.} \end{array}\right) \end{array}$$

So, the *γ*-horizontal cut set of trapezoidal fuzzy number A is [*A*]^*γ*^=[*a* − (1 − *γ*)*α*, *b*+(1 − *γ*)*β*], ∀*γ* ∈ [0,1].

In this paper, we consider the following constraints [19]:

1. Constraint on the number of portfolio assets: in the process of real investment decision-making, there are certain requirements for the number of assets held. Assume that the maximum number of assets held is *M*, then the constraint is ∑_*i*=1_^*n*^sign(*x*_*i*_)=*M*.
2. Investment ratio constraint: the sum of investment ratios for each asset should be 1. Namely, ∑_*i*=1_^*n*^*x*_*i*_=1.

### 4.2. Model Building

As skewness is introduced as a new goal, cardinality constraints and upper and lower bound constraints are added, historical data are replaced by predicted returns, and the specific portfolio model is shown in function (18).

(18) $$\begin{array}{c} \max R\left(x\right)=X^{T}\bar{R}=\sum_{i}^{n}x_{i}\bar{R_{i}},\\ \min V\left(x\right)=X^{T}VX\\ =\sum_{i=1}^{n}\sum_{j=1}^{n}x_{i}x_{j}\sigma_{ij},\\ \max S\left(x\right)=E{\left(X^{T}\left(R-\bar{R}\right)\right)}^{2}\\ =\sum_{i=1}^{n}x_{i}^{3}s_{i}^{3}+3\left(\sum_{i=1}^{n}x_{i}^{2}x_{j}s_{ijj}+\sum_{j=1}^{n}x_{i}x_{j}^{2}s_{ijj}\right)\;\left(i\neq j\right),\\ \text{s.t. }\sum_{i=1}^{n}x_{i}=1,\\ \sum_{i=1}^{n}K_{\min}\leq \theta_{i}\leq K_{\max},\;l_{i}\theta_{i}\leq x_{i}\leq u_{i}\theta_{i},i=1,2,3\ldots ,n,\theta_{i}\in \left\{0,1\right\},i=1,2,\ldots ,n. \end{array}$$

Among them,

 
*n* is the number of available assets
 
*X* is the weight vector formed by the proportion of investment into various assets when each goal achieves the optimal tradeoff
 
*x*_*i*_ is the proportion invested in the ith asset; 12, $\bar{R_{i}}$ 12 is the expected return on the ith asset
 
*σ*_*ij*_ is the return covariance between asset *i* and asset *j*
 
*s*_*i*_^3^, *s*_*ii*_, and *s*_*ijj*_ are skewness and oblique skewness
 
*R*(*x*) is the expected return on the portfolio *x*
 
*V*(*x*) is the return variance of the portfolio *x*
 
*S*(*x*) is the skew of the portfolio *x*
 
*θ*_*i*_ specifies whether an asset *θ*_*i*_ exists in the portfolio
 
*K*_min_ and *K*_max_ are the minimum and maximum number of assets allowed in a portfolio
 
*l*_*i*_ and *u*_*i*_ are the lowest and highest proportion of the investment in asset *i* to the total investment, respectively

The advancement objective of the model is to limit the gamble of the portfolio and expand the normal return of the portfolio and the skewness of the portfolio. Therefore, constraints conclude budget constraints, upper and lower limit constraints, and cardinality constraints. Cardinality constraint ensures that the number of assets in the portfolio is within a certain range where substantial diversified income can be achieved by owning 6 to 15 stocks [20].

The article "Design of Optimum Portfolio Scheme Based on Improved NSGA-II Algorithm" was published in 2022. Journal: Comput Intell Neurosci.

### 4.3. Model Solution

#### 4.3.1. Test Index

Generation distance (GD) and spatial distribution (SS) are selected to test the convergence and accuracy of the algorithm in this paper.

GD refers to the average minimum distance from each point in the solution set *P* to the reference set *P*′, indicating the degree of deviation from the truly optimal boundary. The larger the GD value, the farther away from the true optimal boundary, and the worse the convergence. The specific calculation formula is as follows:

(19) $$\begin{array}{c} \text{GD}\left(P,P^{\prime }\right)=\frac{\sqrt{\sum_{i=1}^{n}d_{i}^{2}}}{n}, \end{array}$$

where *n* is the number of points on the Pareto frontier and *d*_*i*_ is the minimum Euclidean distance between an individual and the real Pareto frontier.

SD indicates the extent of the obtained solution set. The smaller the value of SD, the more homogeneous the solution set. The specific calculation formula is as follows:

(20) $$\begin{array}{c} \Delta =\frac{d_{f}+d_{l}+\sum_{i=1}^{N-1}\left|d_{i}-\bar{d}\right|}{d_{f}+d_{l}+\left(N-1\right)\bar{d}}. \end{array}$$

#### 4.3.2. Test Environment

The hardware environment used in this experiment is Intel Xeon (*R*) CPU ES-2620V4 @ 2.10 GHz, NVIDIA Quadro M4000 GPU, and the running memory is 32G. In addition, the experiment is realized by Matlab simulation. In order to test the performance of the algorithm under different numbers of the target, they are set as 3, 5, and 10, respectively, in the test function. DTLZ (*I*, *M*) represents the spatial distribution of targets in the I dimension, where I is the target dimension and *M* is the number of target objects. The specific parameters are shown in Table 1.

The article "Design of Optimum Portfolio Scheme Based on Improved NSGA-II Algorithm" was published in 2022. Journal: Comput Intell Neurosci.

#### 4.3.3. Test Results

Function (18) was tested with the NSGA-II algorithm and its improved algorithm, respectively, running independently for 10 times, and the test indexes were GD and SD. The experimental results are shown in Table 2.

Table 2 shows that the indicators of GD and SD obtained by the improved algorithm are 2.6509*E* − 05,0.33982, respectively; the GD and SD of the NSGA-II algorithm are 5.7065*E* − 02 and 0.35211, respectively, which shows that the optimization algorithm has the smallest deviation from the real optimal boundary, the best convergence, and the smallest breadth of the solution set. Therefore, the optimized multiobjective algorithm has better convergence, and the distribution of the solution set is more homogeneous.

## 5. Evaluation of Portfolio Design

### 5.1. Scheme Analysis

By taking the fund as an example, if the original capital Y yuan is used for financial investment, then the investment in A, B, C, *D*, and *E* funds can be expressed as

(21) $$\begin{array}{c} Y=A+B+C+D+E,\\ W=aW_{A}+bW_{B}+cW_{C}+dW_{D}+eW_{E}, \end{array}$$

where *Y* is the original fund, *a*, *b*, *c*, *d*, *e* and *W*_*A*_, *W*_*B*_, *W*_*C*_, *W*_*D*_, *W*_*E*_ are the weight and income of funds invested in *A*, *B*, *C*, *D*, *E*, respectively, and *W* is the total income.

### 5.2. Evaluation Indicators

The raw data of this experiment come from the daily trading data of Chinese funds from December 2014 to December 2021, which contains transaction data of various fund prices, each of which consists of time, opening price, maximum price, minimum price, closing price, increase rate, and turnover rate. The daily price data of 10 kinds of funds are selected as experimental data, and only 733 fund price data are selected.

In this paper, the mainstream measurable performance indicators of investment in the current market are adopted, namely, the annual rate of profit, sharp ratio, and forecast rate of profit [21, 22].

(1) Annualized rate of profit
The annualized rate of profit is a measure of the profitability of investors during the investment period of one year
  (22) $$\begin{array}{c} \text{Annualized rate of return }=\frac{\text{Income}/\text{capital}}{\text{Investment days}/365}\times 100\text{\%.} \end{array}$$
(2) Sharp ratio
Sharp ratio is a standardized index to evaluate the fund performance
  (23) $$\begin{array}{c} \text{Sharpe Ratio}=\frac{E\left(R_{P}\right)-R_{f}}{\sigma_{P}}. \end{array}$$
where *E*(*R*_*P*_) represents the expected return rate of risk asset portfolio; *R*_*f*_ is the risk-free rate of return, which can be replaced by the interest rate of 10-year Treasury bonds, that is, 2.85%; *E*(*R*_*P*_) − *R*_*f*_ is the risk premium. When the Sharp ratio <0, the return on investment is not as good as the return on Treasury bonds.
(3) Predicted rate of profit
The estimated pace of profit from the venture, otherwise called the speculation benefit rate, alludes to the proportion of the absolute yearly net gain of the speculation plan to the all speculation of the plan in a year subsequent to arriving at the planned limit of creation
  (24) $$\begin{array}{c} \text{Predicted rate of profit}=\frac{\text{Annual pre}-\text{tax profit }}{\text{Total investment of project}}\times 100\text{\%.} \end{array}$$

The article "Design of Optimum Portfolio Scheme Based on Improved NSGA-II Algorithm" was published in 2022. Journal: Comput Intell Neurosci.

### 5.3. Analysis of Results

The multiobjective portfolio model algorithm mentioned above is iterated for 50 times to get the weight of each industry coefficient in the scheme of the portfolio. The results are shown in Table 3.

According to a certain capital, the annual return, investment profit, and Sharp ratio within 2 years are calculated, respectively, according to the portfolio scheme obtained by NSGA-II and its optimization algorithm, as shown in Table 4.

From the data in the table, it can be seen that the annualized profits of the portfolio scheme within two years obtained by NSGA-II and its optimization algorithm are 37.60% and 41.25%, respectively. The predicted profits on investment are 63.24% and 70.08%, respectively; the Sharp ratio of the two portfolio schemes is greater than 0, which indicates that the income of investment exceeds that of the Treasury bonds. Therefore, the portfolio scheme obtained by the multiobjective optimization algorithm is the best.

## 6. Conclusion

Based on the portfolio theory, this paper introduces the t-SNE optimized NSGA-II algorithm to establish a multiobjective portfolio model for the multiobjective optimization of portfolio investment in the financial industry, where the expected return, risk, skewness, and other indexes of securities are quantified, and the solving algorithm of the model is evaluated by the generation distance and spatial distribution. The evaluation results show that the annualized profits of the portfolio scheme obtained by the optimized algorithm are 41.25%, the predicted profits on investment are 70.08% within two years, and its evaluation of performance is higher than that of the NSGA-II algorithm.

The article "Design of Optimum Portfolio Scheme Based on Improved NSGA-II Algorithm" was published in 2022. Journal: Comput Intell Neurosci.

## Figures and Tables

**Figure 1:** Advantages of NSGA-II algorithm.

**Figure 2:** Flow chart of NSGA-II algorithm. The fundamental advances are as per the following [15, 16].

**Figure 3:** Algorithm optimization based on *t*-SNE.

**Figure 4:** Membership function of fuzzy number A.

**Table 1:** Test parameters.

Name	Expression	Value
Species size	Species size	500
Evolutionary algebra	Generation	10000
Variation probability	Pm	0.1
Cross probability	Pc	0.9
Data dimension	*V*	12
Analog binary crossover parameter	*L*	50
Polynomial variation parameter	*U*	5

**Table 2:** Model test results.

Test categories		NSGA-II	Improved NSGA-II
Generation distance	Standard	5.7065*E* − 02	2.6509*E* − 05
	Error	2.1500*E* − 03	4.9200*E* − 05
Spatial distribution	Standard	0.35211	0.33982
	Error	0.00977	0.0103

**Table 3:** Weight of portfolio.

Serial number	NSGA-II algorithm	Optimization algorithm
1	0.265	0
2	0.102	0.196
3	0.249	0.185
4	0	0
5	0.127	0.287
6	0.164	0.234
7	0	0
8	0.045	0.060
9	0	0
10	0.048	0.038

**Table 4:** Performance evaluation.

	NSGA-II algorithm	Optimization algorithm
Annualized rate of profits/%	37.60	41.25
Forecast rate of profits/%	63.24	70.08
Sharp ratio/%	74.26	93.65

## Data Availability

The dataset can be accessed upon request.
